# Aerodynamic Analysis and Training Research of an S-Shaped Arc Ball Based on Hydrodynamics

**DOI:** 10.1155/2022/1088906

**Published:** 2022-08-25

**Authors:** Pinxin Si

**Affiliations:** Guilin University of Aerospace Technology, Guilin, Guangxi, China

## Abstract

The aerodynamic characteristics of S-shaped arc ball, such as poor combat performance and low intelligence, are studied and analyzed. In this paper, the aerodynamic analysis model of S-shaped arc soccer intelligent algorithm is established, and the dynamic tracking model of Soccer Tactics Based on fluid dynamics search algorithm is designed. The data information is collected from many aspects, such as the position of the players, the change of the arc ball movement, the trajectory of the football movement, and tactical flexibility. The results show that Benn's algorithm can start the layout mechanism effectively. It has high feasibility and accurate algorithm accuracy and can effectively improve the aerodynamic layout performance of the system. The aerodynamic analysis and training optimization method of the S-shaped arc ball based on ant colony optimization has sped up the intelligent training system of Chinese football tactics.

## 1. Introduction

Up to now, the fixed tactic is the main process of the physical education in Chinese universities, and the multitactic integration mode of the main members is the auxiliary [1]. In recent years, with various information in China, the reform of the football system has been brought about. The tactic teaching methods such as intelligent football tactics, multitactic combination, key point taking method and so on, For the new teaching of football tactics and the mode of football optimization cooperation in colleges and universities on a large scale [2]. Therefore, football sports intelligence part of the current [3]. Achieve the best effect of football practice according to their own actual experience structure and their own advantages in the daily practice. In this context, the aerodynamic system of the S-shaped arc ball based on a deep learning intelligent algorithm is proposed.

The innovation of this paper is to improve the ant colony optimization search algorithm. On this basis, the algorithm is applied to the aerodynamics analysis of the S-shaped arc ball in football, so that the station information of each football tactic and the physical characteristics of players can be fully utilized to achieve the overall approach through real-time dynamic tracking. The similarity degree between factor and the degree of consistency between the expected indexes are described quantitatively. The order of the influence degree of training system indexes is completed by the quantitative index, and the factors affecting the aerodynamics of the S-shaped arc ball can be analyzed in a customized way.

Section 2 constructs the tracking training model of the S-shaped arc ball based on the ant colony optimization search algorithm.  Section 3 tests the aerodynamic analysis and training model of the S-shaped arc ball, and Section 5 concludes the results.

## 2. State of the Art

With the connotation and manifestation of the core quality of physical education and health discipline, this paper studies and discusses the significance and measures of implementing the fundamental task of “building morality and cultivating people” and the educational concept of “health first” from the three aspects of sports ability, healthy behavior, and sports morality. At the same time, it deeply analyzes the practical and cognitive problems existing in the implementation of the new curriculum standard [4]. The significance of intelligent physical education teaching reform and the latest research and application results of the educational informatization application community project of the Ministry of Education. From the teaching mode of intelligent physical education, guidance and evaluation, virtual simulation experiment and theory of sports skills. VR intelligent sports teacher, functional sports homework tracking system. The visual evaluation of basic motor skills and other aspects shared the new exploration of intellectual sports on the implementation of the new curriculum standard [5]. Scientific research on athletes' sports and preparation is constantly developing. This development is mainly based on the continuous in-depth. Athletes' physiological and competitive ability, in order to improve athletes' competitive performance [6]. With the improvement of our knowledge of physical stress, today's training theory researchers and sports researchers explain the most basic concepts of training [7].

The core of training theory is to establish a structured system of training according to the training activities of different sports and athletes' physiological, psychological, and sports characteristics, so as to adjust the training adaptation process and guide the specific training [8]. This adjustment and guidance process can be better understood by understanding bioenergetic functions (i.e., how the body supplies energy). Bioenergetic characteristics are used to meet the physical needs of different body movements [9]. Coaches should understand the bioenergetic characteristics of physical activities and sports, as well as the influencing factors of the specific time arrangement of training stimulation for physical adaptation, which will make it more possible to formulate an effective training plan. Athletes complete a specific goal and pass the training system. The purpose of training is to improve athletes' competitive ability, so as to improve sports performance [10]. Training is a systematic project, which involves many variables of physiology, psychology, and sociology. During this period, the training should follow the basic principles of step-by-step and differential treatment. In the whole training process, the physical and psychological quality of athletes can be shaped to meet some strict task requirements [11].

According to the tradition of ancient Olympic movement, integrate excellent physical ability with spiritual realm and noble sentiment. Physical excellence means diversified and harmonious development. Athletes need to have exquisite and diverse skills, cultivate positive and stable psychological quality, and maintain the best health [12]. Athletes should learn to deal with the great pressure in training and competition. Excellent physical ability must be realized through training practice, well-planned training courses, and training methods with scientific basis [13]. Based on the ant colony optimization algorithm of a multidimensional data information factor, scholars selected three indicators related to the impact of football players and tactical training system and proposed an S-shaped arc ball aerodynamic system based on players' training characteristic parameters and ant colony optimization search algorithm, through the research on tactical selection, gait analysis and detection, and the position of the station [14].

The aerodynamics of the S-shaped arc ball of football does not involve the analysis of the deep learning intelligent algorithm based on hydrodynamics theory and football movement data [15]. Whether beginners or professional athletes, the most important thing is to set practical training goals. Training objectives should be designed according to personal ability, psychological characteristics, and social environment. Some athletes train in order to win the competition or improve their performance, while others are in pursuit of acquiring sports skills or further improving their biological movement ability. No matter what the target is, it should be as accurate and measurable as possible. Whether it is a short-term plan or a long-term plan, it should be set before the training starts, and the specific details of the process of achieving the goal should be clear. The final moment to achieve these goals is often a major game.

## 3. Methodology

### 3.1. Deep Learning Intelligent Algorithm in the Aerodynamic Analysis Model of the S-Shaped Arc Ball

In the process of studying the aerodynamics of the S-shaped arc ball, in order to realize the stability of the analysis model through the deep learning intelligent algorithm and fluid mechanics theory, the team adopted the improved ant colony optimization search algorithm to realize the intelligent detection and analysis of the daily S-shaped arc ball in the aspect of aerodynamics [16]. There are many ways to classify physical sports skills. In addition to the traditional classification method, which divides sports using biological movement ability, the classification standard is also a widely accepted classification method [17]. Biological movement ability includes strength, speed, endurance, and coordination ability. Although it is very practical to use biological movement ability to classify sports, coaches often use some other classification. The classification method is to divide motor skills into cyclical skills, aperiodic skills, or aperiodic combination skills (in this paper, it refers to the gait signal of football players and the detection node of S-shaped arc ball movement). The coupling analysis of gait dynamic characteristics and key point selection, as well as the vector processing analysis of multiple coupling combinations [18], can achieve the signal optimization and analysis processing of the whole football movement control.  Figure 1 illustrates the basic principle of ant colony optimization.

This deep learning intelligent algorithm determines the predicted position of football movement from the total aerodynamic analysis process of the S-shaped arc ball and finds the group with high similarity between the S-shaped arc ball and the dynamic gait signal of football players and then the probability. High level competitive ability carefully planned, systematic period, athletes constantly adjust their physiological functions to meet the special requirements of special sports. The higher the adaptability of athletes to the training process, the more they can play a high level of sports potential. Only when athletes follow the following order can they improve their sports performance. The stimulation (load) that athletes need to increase must be greater than the improvement of training performance on the basis of adaptation. If the stimulation is too excessive or too complicated, athletes will not be able to adapt and maladjustment will occur. These changes of training stimulation refer to the changes of training elements to maximize the athletes' adaptation to the training plan [19]. We can realize the unique gait information analysis record and the coupling analysis of the soccer S-curve ball under the condition of optimized ant colony optimization. The more the accumulated soccer players' dynamic gait data and soccer S-curve ball movement data, the more the process, which is also in line with the characteristics of the deep learning intelligent algorithm [20]. The above is the basic principle of ant colony optimization S-shaped arc ball aerodynamic analysis and data processing. The analysis results of its aerodynamic three-dimensional space motion process are shown in Figure 2, where *Z* represents different search mechanisms, *P* is the location information, and *v* is the speed information. The common S-shaped arc ball aerodynamic analysis method, accurate tactical analysis, and data correction were compared, so as to give full play to the practical value of football players' tactical training process.

### 3.2. The Realization Steps of the Aerodynamic Analysis Model of the S-Shaped Arc Ball Based on Hydrodynamics

The technology may bring significant changes to the sports. To watch the game video and manually record the actions of a single player—including the number of passes and shots, the place where the actions occur, and whether they are successful or not. This method not only is very time-consuming but also has problems. Players often spend countless hours training to improve their skills so that they can become more competitive in sports events such as basketball. In order to help players improve their skills, systems have been developed that track players' performance during training or games and then provide feedback indicating performance. This feedback can then be evaluated to help the player improve his skills. Researchers have made some achievements by taking advantage of the latest progress in the fields of computer vision, deep learning, and artificial intelligence.

Based on the latest progress of artificial intelligence and deep learning, an artificial intelligence model is used to detect athletes' limbs and posture. Tracking where the ball lands in the hoop while shooting may present a variety of challenges that may limit the effectiveness of systems that attempt to evaluate projection performance. As an example, since the shooter is on one or the other side of the court, many basketball shots are usually at a nonorthogonal angle to the backboard (and the corresponding hoop). Shooting from different angles often leads to different shooting positions in the basketball circle. Specifically, based on the theoretical framework of the ant colony optimization search algorithm, the hydrodynamics analysis process of the S-shaped arc ball is shown in Figure 3, where *S* represents different position states and *E* represents different energy states.

Next, the S-shaped arc ball is analyzed and processed from the perspective of hydrodynamics. The implementation steps are shown in Figure 4, where *S* represents different position states and *E* represents different energy states.

For the two different ways, we need to complete the data analysis and processing through the following steps.

Step 1. We need to initialize the parameters. First, set the time *t* = 0, NC = 0:

(1) $$\begin{array}{c} \tau_{ij}\left(\text{NC}t\;\max\right)=\text{const}+C, \end{array}$$

where *C* is the constant and Δ*τij*(0) = 0.

Step 2. We need to set the number of cycles:

(2) $$\begin{array}{c} \text{NC}=\text{NC}+1. \end{array}$$

In this step, the index number of the taboo table in the signal processing process of S-curve ball data is *k* = 1. The number of key nodes in the detected position is

(3) $$\begin{array}{c} k=k+1. \end{array}$$

Step 3. After modifying the tabu list pointer, that is, after selecting it, we will move the detected aerodynamic signal of the S-shaped arc ball to the new element set and move the element to the detected tabu list set. If the elements in the collection are not traversed completely, jump to the next step to realize the loop; otherwise, execute the last step.

Step 4. Formulas (2) and (3) represent the advantages and disadvantages of the aerodynamic signal processing degree of the detected S-shaped arc ball.

Step 5. After updating the amount of information, if the end condition is satisfied, the cycle will end and the program calculation results will be output. Otherwise, the tabu list will be cleared, and jump to the second step. This is the basic implementation process of dynamic gait tracking and tactical key point decision processing ant colony optimization. In the pheromone update phase, we use the adaptive pseudorandom ratio to select the next detected football gait signal *F* (*j*) as the pheromone:

(4) $$\begin{array}{c} F\left(j\right)=\arg\;\max\left\{\tau \;\left(i,j\right)\eta \;\beta \;\left(i,j\right)\right\},q\leq q0. \end{array}$$

## 4. Result

### 4.1. Experimental Design of the Aerodynamic Analysis Model of the S-Shaped Arc Ball Based on Hydrodynamics

When analyzing lower league or grassroots games, a process used to evaluate projection performance enables the system to capture shots using one or more cameras and then determines the athlete's trajectory and shooting location. Then, the system can use the trajectory of shooting to determine the position of athletes on the sports field. Once the position of the athlete and the origin of the movement are determined, the system can determine the position of the front of the hoop relative to the position of the athlete. In the game, the deep neural network is also trained to track individual players in the whole game video and collect personal performance data. Tracking players can help understand the relationship between players' positions and others—this information is very important when analyzing team sports coordination. The algorithm process is shown in Figure 5.

In this model, the different gait modes of different football players and how to analyze whether the football gait of the detected person meets the best requirements of relevant fluid dynamics are mainly based on the intelligent combination mode; the aerodynamics analysis and tactical switching prediction of the S-shaped arc ball for a local specific target are realized. The characteristic of this intelligent comprehensive evaluation method filters the gait characteristics of the whole football player group in advance but carries out intelligent processing according to the automatic association analysis system, so as to realize the innovation of the method for the research of S-shaped arc ball aerodynamics.

Therefore, football S-shaped arc ball aerodynamic information big data based on fluid mechanics, the aerodynamic signal of different players' football S-shaped arc ball, and the gait information data of the target to be analyzed are compared in pairs, so as to achieve multilevel comparative analysis. By unified orthogonalization, the initial weight required by the optimized ant colony optimization algorithm and the prediction of normal soccer S-shaped arc ball aerodynamic data are the minimum threshold. Through the above process, we can find that, compared with the traditional processing method.

### 4.2. Aerodynamic Model of the S-Shaped Arc Ball

The detection data of other common detection methods of S-shaped arc ball aerodynamics are shown in Figure 6, and the signal data of key nodes detected in the experiment based on the deep learning intelligent algorithm are shown in Figure 7.

Up to now, there is no specific standard for the evaluation of football training effect. Therefore, this study takes two football S-curve balls with different trajectories as two groups of tracking research subjects and takes a random player (the player's football level is general, and the process is that the actual football performance is between 30% and 70% of the team performance ranking, randomly selected by random number) as the control experiment object; one player's football competitive level at the beginning is lower than medium (football actual performance ranking is beyond 80% of the team), and the other player's football level is lower than high (football actual performance ranking is within 20% of the team). It is found that in the comprehensive performance of the new football competition, the two players have a great improvement in the prediction of the S-shaped arc ball, and the actual performance of one player has been promoted from beyond 80% to less than 30%. Another player from the actual performance ranking in professional within 20% to 11%. Therefore, the experimental results show that the aerodynamic analysis and training model based on the ant colony optimization search algorithm and fluid dynamics can accurately compare and analyze the current state of the S-shaped arc ball. The player who is engaged in a certain goal is affected by the S-curve ball. Therefore, the experimental results show that the aerodynamic analysis method based on the ant colony optimization search algorithm and fluid dynamics can be applied to the real-time detection and processing of professional football tactics.

## 5. Conclusion

The reform of football training system and tactic teaching mode is imperative. Based on this, this paper adopts the deep learning intelligent algorithm based on multicorrelation factors and the hydrodynamics analysis method. Firstly, three characteristic parameters related to the aerodynamic influence index of the S-shaped arc ball are selected. Secondly, through the research on the selection of rotation, the analysis of movement state, and the situation of movement position, the S-shaped arc ball aerodynamic model is clearly defined. Finally, the deep learning intelligent algorithm is used to analyze the features of the screening results. The experimental results show that the training system position and the aerodynamic characteristics of S-shaped arc ball achieve close to the integrity of the players and can improve the football actual combat level of the players. However, this paper only focuses on the aerodynamic analysis and training system construction of the S-shaped arc ball and does not take into account the potential impact of the overall coordination of football tactics.

## Figures and Tables

**Figure 1:** The basic principle of ant colony optimization.

**Figure 2:** 3D space motion analysis process of aerodynamics.

**Figure 3:** Analysis results based on the ant colony optimization search algorithm.

**Figure 4:** Analysis results based on fluid mechanics and intelligent algorithms.

**Figure 5:** Training model and process based on the deep learning intelligent algorithm.

**Figure 6:** Experimental test results of common methods.

**Figure 7:** The method proposed in this research.

## Data Availability

The data used to support the findings of this study are included within the article.
